The article "Sequence Fusion Algorithm of Tumor Gene Sequencing and Alignment Based on Machine Learning" was published in 2021. Journal: Comput Intell Neurosci.

# Sequence Fusion Algorithm of Tumor Gene Sequencing and Alignment Based on Machine Learning

**DOI:** 10.1155/2021/9444194

**Published:** 2021-12-31

**Authors:** Chao Tang, Ling Luo, Yu Xu, Guobin Chen, Li Tang, Ying Wang, Yongzhong Wu, Xiaolong Shi

**Affiliations:** ^1^Radiation & Cancer Biology Laboratory, Radiation Oncology Center, Chongqing Key Laboratory of Translational Research for Cancer Metastasis and Individualized Treatment, Chongqing University Cancer Hospital & Chongqing Cancer, Institute & Chongqing Cancer Hospital, Chongqing 400030, China; ^2^The Department of Internal Medicine, Chongqing University Cancer Hospital & Chongqing Cancer, Institute & Chongqing Cancer Hospital, Chongqing 400030, China; ^3^College of Bioengineering, Chongqing University, Chongqing, China; ^4^Chongqing Key Laboratory of Spatial Data Mining and Big Data Integration for Ecology and Environment, Chongqing Finance and Economics College, Chongqing 401320, China

## Abstract

With the rapid development of DNA high-throughput testing technology, there is a high correlation between DNA sequence variation and human diseases, and detecting whether there is variation in DNA sequence has become a hot research topic at present. DNA sequence variation is relatively rare, and the establishment of DNA sequence sparse matrix, which can quickly detect and reason fusion variation point, has become an important work of tumor gene testing. Because there are differences between the current comparison software and mutation detection software in detecting the same sample, there are errors between the results of derivative sequence comparison and the detection of mutation. In this paper, SNP and InDel detection methods based on machine learning and sparse matrix detection are proposed, and VarScan 2, Genome Analysis Toolkit (GATK), BCFtools, and FreeBayes are compared. In the research of SNP and InDel detection with intelligent reasoning, the experimental results show that the detection accuracy and recall rate are better when the depth is increasing. The reasoning fusion method proposed in this paper has certain advantages in comparison effect and discovery in SNP and InDel and has good effect on swelling and pain gene detection.

## 1. Introduction

With the rapid development of high-throughput sequencing and gene chip technology, DNA sequence variation detection and chip expression have become the current research hotspots. In the massive data generated by sequencing, it is found that there is a correlation between structural variation and gene expression. With the increasing amount of human genome data, Single Nucleotide Polymorphism (SNP) and Insertion and Deletion (InDel) variants will be found more and more.

In view of the more than 60 existing kinds of comparison software, Bowtie 2 [1], Burrows–Wheeler Aligner (BWA) [2], HISAT2 [3], and Subread [4] are used more frequently and more effectively than other software tools. This paper focuses on the comparative study of these four kinds of software and, through relevant comparative analysis, studies the fusion of BAM files produced by the four kinds of software, so as to produce the best BAM files.

NGS technology has high throughput; that is, the amount of data sequenced at one time is large, the read data can reach tens of millions, and the sequencing depth is relatively deep, and many exons can reach 1,000x. Compared with the traditional SNP discovery method, it has obvious advantages and relatively large amount of mining information. However, with the emergence of a large amount of high-throughput data, some sequencing sequences will also lead to sequencing errors, and the sequencing quality, systematic errors, and random errors will also increase, which will also lead to the inevitable problems such as wrong suggestions caused by the analysis of test results. For example, Copy Number Variations (CNV), Insertion and Deletion (InDel), and Structural Variation (SV) in genetic variation make the analysis unpredictable. There are many existing SNP detection processes, but the mainstream SNP Calling software for SNP detection, such as VarScan 2 [5], GATK [6], BCFtools [7], and FreeBayes [8], also has its own detection advantages, and the detection structures of various software are the same as those of comparison software. SamTools, BCFTools, and GATK use Bayesian statistical models. Such models perform well in the analysis of diploid genomes but may be hindered by extremely deep coverage or data sets with low allele scores. In fact, a recent comparison of variation detection tools for tumor subclonal analysis [9] found that VarScan 2 showed obvious differences when the sequencing depths required for accurate identification of variants were 100x, 250x, 500x, and 1,000x, respectively [10]. Different SNP detection software has different detection results, so it is necessary to comprehensively utilize the advantages of the above software to generate a detection method based on multidetection software fusion.

### 1.1. Burrows–Wheeler Transformation Technique

Assume that Σ={*A*, *C*, *G*, *T*} is the alphabet that makes up the sequence and is a symbol smaller than the lexicographic order of all characters in it. Given a string *S*=*a*_0_*a*_1_,…, *a*_*n*_, where *a*_*n*_=$, so that *S*[*i*]=*a*_*i*_ represents the *i*-th letter, *S*[*i*, *j*]=*a*_*i*_,…, *a*_*j*_ is a subsequence of *s*, and *S*_*i*_=*S*[*i*, *n* − 1] is a suffix of *S*. *S* is the Burrows–Wheeler transformation (BWT) structure which is the result of n-step right-shift operation on *S*, one character at a time, and a matrix array of *n* rows is obtained. Each row in the array is a result of *S*-right-shift operation, and the string before the $ character is the suffix corresponding to the row. After the matrix is established, the suffix of each row in the matrix is sorted according to the dictionary order and then rearranged to get the final conversion array. The characters in the last column of the matrix can be combined in turn to get the converted string sequence. The following calculation of BWT(*S*) for a given string *S* includes three basic steps:

  Step 1: append a special symbol $ to the end of *S*, which is smaller than any symbol in *S*.
  Step 2: construct the *M* matrix, the first row of which is equal to *S.* Row 2 of the *M* matrix is cyclically shifted one bit to the right of row 1 of the *M* matrix (*S* value). Row 3 of the *M* matrix is cyclically shifted one bit to the right of row 2 of the *M* matrix, and this is repeated until reaching row *n*. Through the observation of the matrix, it can be found that when the *n*th row of the matrix shifts to the right by one bit, the first row *S* will be obtained again, which means that the sequence cyclic shift is executed until the *n*-th row, just completing a rotation of sequence *S*.
  Step 3: construct the converted text *S* = BWT(*S*) by taking the last column of the *M* matrix.

Note that every column of the *M* matrix, that is, the converted text *S*, is an arrangement of *S*$.

**Example 1 .**

*S* = “ACGTACAAAT” is used to illustrate the conversion process. The specific operation steps are as follows:

  Step 1: *S* = “ACGTACAAAT” is used to illustrate the conversion process, and a character $ is added after *S* to form *S*$, that is, *S* = “ACGTACAAAT $,” the first behavior of the *M* matrix “ACGTACAAAT $.”
  Step 2: the second row “CGTACAAAT$A” is obtained by cyclically shifting *S* to the right once to form the second row of *M* matrix, and the third row “GTACAAAT$AC” is obtained by cyclically shifting the second row of *S* to the right once. The *n* − 1 row of *S* is cyclically shifted to the right once (*n* is the length of *S*), and the *n*th row of *M* matrix, that is, the last row “$ACGTACAAAT,” is obtained, and finally the *M* matrix is formed. Then the *M* matrix is sorted (the principle of $ < *A* < *C* < *G* < *T*), and the *M* matrix is obtained.
  Step 3: take the last row of *M* matrix, namely, BWT(*S*), and the specific effect is shown in Figure 1.

Figure 1 shows the structure construction process of string *S* = “ACGTACAAAT$.” String *S* is obtained by 10 rounds of circular right shift operation, in which the last letter of each row in the matrix is combined to obtain the new string = “TCAT $AAACAG” after BWT conversion. *S*(*i*) and *i* in Figure 1 are described in FM-index. The last column and the original sequence are not reduced in number, which can achieve lossless compression effect. There are many identical strings on $\hat{S}$. If $\hat{S}$ is compressed by other compression methods, it can also achieve good results.

### 1.2. Based on Hash Indexing Technology

The method based on hash index is often used to query and match in large databases and can also achieve accurate matching in DNA sequences. By querying the index relationship of sequencing sequences in reference genome, we can detect whether sequencing sequences exist in DNA sequences. This kind of technology is explained as follows:

  Step 1: hash table creation.

In DNA sequence, it is composed of four basic units: *A*, *C*, *G*, and *T* (*N* is not taken as the statistical range). The continuous sequence with length *K* is called “seed,” and there are 4*K* kinds of sequences. A hash table is established for 4*k* seed sequences. Because binary has certain advantages in expressing characters *A*, *C*, *G*, and *T*, it can uniquely identify DNA sequences, as shown in the following formula:

(1) $$\begin{array}{c} f\left(x\right)=\left\{\begin{array}{c} 00\begin{array}{c} x={\;}^{\prime \prime }A{\;}^{\prime \prime }, \end{array}\\ 01\begin{array}{c} x={\;}^{\prime \prime }C{\;}^{\prime \prime }, \end{array}\\ 10\begin{array}{c} x={\;}^{\prime \prime }G{\;}^{\prime \prime }, \end{array}\\ 11\begin{array}{c} x={\;}^{\prime \prime }T{\;}^{\prime \prime }. \end{array} \end{array}\right. \end{array}$$

Seed *W* can be expressed in a unique way, remember *V* (*W*), as shown in the following formula:

(2) $$\begin{array}{c} V\left(w\right)=\overset{k}{\underset{i=1}{\sum }}4^{i-1}f\left(x_{i}\right). \end{array}$$

  Step 2: association of the reference sequence hash table.

Human DNA sequence can be divided into 23 pairs of chromosomes, each pair of chromosomes has a large number of DNA sequences, and the chromosome sequence is represented by *D* = {chr1, chr2,…, chr23}. The length of sequential seed *w* of DNA sequence decomposition in each chromosome is set to *K* = 4 or *K* = 8, or even higher, every shift of one bit from the beginning of the sequence to the end of the sequence. If the sequence length is *L*, then the sequence has *L* − *k* + 1 seeds. For the sequence *N* (*N* = 1, 2,…, *N*) of the “seed” and the position number *L* (*L* = 1, 2,…, *L*) in the sequence, the hash table (*N*, *L*) of the “seed” is established. If the hash table is established for *S* = “ACGTACAAAT,” the procedure is as follows:

Take sequence *S* = “ACGTACAAAT,” *k* = 2, as an example, as shown in Table 1.

  Step 3: the alignment sequence can also decompose the seeds with length *K* and then refer to the hash table of the established reference sequence to find the corresponding position information.

For example, the query “TAC” is decomposed into “TA” and “AC” hash tables corresponding to (1, 4), (1, 1), and (1, 5), respectively. The positions (1, 4) and (1, 5) are correlated, so the position of “TAC” in *S* is 4.

The location query algorithm based on hash table indexing technology, if there are sequencing errors in sequencing sequences, SNV, InDel, and so forth, will lead to matching errors or sequence matching to other locations. Biological alignment software, such as MAQ [11], RMAP [12], ZOOM [13], and so forth, indexes sequencing sequences, while others index reference sequence databases. Delete the “seeds” in the hash table whose frequency is lower than the set threshold. Because the length of reference genome is fixed, indexing reference sequences can improve the efficiency of sequence alignment. Generally, the index can be stored in advance, and the sequencing sequence can be decomposed into *K* seeds to match the established hash table.

### 1.3. Suffix Tree Detection Algorithm

#### 1.3.1. Suffix Tree [14]

Let Σ be *n* sequences in a finite DNA sequence, and the suffix tree *S* is a directed tree with roots, where *n* leaves are exactly numbered 0 to *n* − 1, corresponding to each suffix of *S*. Each internal node has at least two child nodes, and each edge is marked with a nonempty substring of *S*. Neither edge other than the same node is allowed to have an edge label beginning with the same character. For any leaf *I*, the concatenation of edge tags on the path from root to leaf *I* accurately spells out the *S* suffix starting at position *I*, that is, substring *S* [*i*,…,*n*]. Add a unique terminator $ ∉ Σ at the end of the string to ensure that the suffix is prefixed to any other suffix. The edges of the suffix tree join those nodes in the tree which have only one character, so that each internal node in the suffix tree will have at least two child nodes. In this way, redundant nodes are reduced, thus saving the construction time and space of suffix tree. Each path from the root node to the leaf node in the suffix tree represents a suffix subsequence, and the value in the last leaf node represents the starting position of this subsequence. When they have the same internal node, they have the same common prefix.  Figure 2 shows the suffix tree transformation process for the reference genome *S* = “ACGTACAAAT.”

For the reference genome *S* = “ACGTACAAAT$,” each subsequence is on the leaf node of the suffix tree. In the target sequence, $ still indicates that the sequence and its suffix terminate, occurring only once at the end of the sequence or at the end of the subsequence. Similar to a dictionary tree, if the sequence in which a suffix tree is constructed contains *K* characters, then the suffix tree has *K* + 1 branches (including termination symbols) from the root node. In Figure 2, the DNA sequence *S* has only four characters, *A*, *C*, *G*, and *T*, plus a branch of the terminator, so there are five branches from the root node. There is only one suffix starting with character *G*, and there are no other branches. Leaf nodes need to be stored in the suffix tree, as well as the path of edges.

The suffix array can be obtained by transforming the suffix tree. The suffix array is arranged according to the dictionary order, and the initial position information of the arranged suffix tree establishes one-to-one correspondence with the reference gene sequence. The suffix array *A* of string *S* is an array of integers in the range from 0 to *n*, specifying the dictionary order of *N* + 1 suffixes of string $; that is, SA[0], SA[1],…, SA[*n*] is the ascending sequence of suffixes of *S*$ as shown in Figure 3. Suffix arrays require 4*n* (8*n* on 64 bits) bytes of memory, so they are memory inefficient and cannot be used for large sequences.

### 1.4. FM-Index Technology

FM-index [15] is a full-text string index based on BWT compression, somewhat similar to a suffix array. It consists of a BWT count array *C*[*p*] and an occurrence table Occ(*p*, *k*). For each character *p* in the letter, the count array *C*[*p*] is defined as the number of occurrences of fewer characters in the string, and Occ(*p*, *k*) is defined as the number of occurrences of character *p* in BWT[0,…, *k*]. The main difference between FM-index and suffix arrays is the way the search is performed. FM-index searches for strings backwards, whereas, in suffix arrays, string matching goes forward. The following is an example of an FM-indexed data structure with string *S* = “ACGTACAAAT”:

  Step 1: constructing *M* matrix, sequencing sequences *S* and $, performing sequences of rotating columns on *S*$, and then performing row sorting with *M* matrix to obtain *M*′.
  Step 2: establish a corresponding relationship between the rows in the *M*′ matrix and the rows in the *M* matrix, and remember *B*[*i*] in the last column in *M*′. *M*′ and *S* can be restored by the inverse process of BWT.
  Step 3: create an array where Oc($), Oc(*A*), Oc(*C*), Oc(*G*), and Oc(*T*) represent the row number of the first occurrence of the first column of the matrix. Occ(2,*G*) represents the number of occurrences in the last column, and the FM-index transformation process is shown in Figure 4. FM-index and suffix array have some similarity. The first column of *M*′ matrix is denoted as *F*[*i*], and the last column of matrix is mapped to *F*[*i*] as LF[*i*], which is realized by the combination of Oc and Occ arrays above, and denotes LF[*i*] = Oc[*L*[*i*]] + Occ[*L*[*i*],*i*]. In the search process, it is expressed by setting the search scope formula:

(3) $$\begin{array}{c} \left\{\begin{array}{c} L=Oc\left[F\right]+Occ\left[L,F\right],\\ H=Oc\left[F\right]+Occ\left[H+1,F\right]-1, \end{array}\right. \end{array}$$

where *F*∈ {*A*, *C*, *G*, *T*}, *L* = 0, *H* = *N* − 1 is the initial value, *H* − *L* − 1 is the number of times character *F* appears, and *S* [*L*, *H*] is the position of the character, as shown in Figure 4.

The following is an example to verify the above method, the number of times *L* = “TAC” appears in *S* = “ACGTACAAAT,” and the operation is as follows:

  Step 1: look forward from the back of string *L*, setting two variables, *R* and *H*, to indicate the minimum position and the maximum position, and *R* = 0 and *H* = 10 to indicate the position from 0 to 10. The last character in *L* is “*C*.” Looking for the position of “*C*” through *Oc* and Occ, it is determined that *L* = *Oc*[C] + Occ[0, C] = 6 + 0 = 6 and *H* = *Oc*[C] + Occ[10 + 1, C]  − 1 = 6 + 2 − 1 = 7. It can be seen that *H* − *L* + 1 = 2 means that there are two “*C*” in *S* string, and the positions are *S*[6] and *S*[7], respectively.
  Step 2: calculate new *L* and *H* from the second rightmost character “*A*,” where *L* = 6 and *H* = 7. *L* = *Oc*[A] + Occ[0, A] = 1 + 2 = 3, *H* = *Oc*[*A*] + Occ[8, A] − 1 = 4, and *H* − *L* + 1 = 2 mean that “AC” occurs twice in the *S* string, and the positions are *S*[3] = 4 and *S*[4] = 0, respectively.
  Step 3: finally, look for “*T*.” At this time, *L* = 3 and *H* = 4 calculate *L* and *H* again. *L* = *Oc*[T] + Occ [3, T] = 1, *H* = *Oc*[T] + Occ[4, T] − 1 = 10 and *H* − *L* + 1 = 10 − 10 + 1 = 1 indicate that “TAC” occurs once in the *S* string, and the position *S*[10] = 3.

This method can be used to find the number and position of characters in the string, and the algorithm complexity is *O*(*n*). In the software of DNA sequence comparison, the advantage of FM-index algorithm is that it can save memory and realize sequence alignment on personal computer.

In the second part of the article, we use hash index, Burrows–Wheeler transform, suffix tree, and suffix array, as well as FM-index to DNA sequence alignment algorithm.

Hash index technology is equivalent query; hash index has an absolute advantage, but the premise is that there are not a large number of duplicate key values. If there are a large number of duplicate key values, the efficiency of hash index is very low because of the so-called hash collision problem. The comparison of algorithm performance query effect is mainly that a large amount of storage space is needed when establishing index space. The time complexity of query is *O*(*n*), while the position join after query needs *O*(*n∗m*).

Burrows–Wheeler transform is a full-text indexing method, which is a search and compression method based on characters. If the original string has several substrings that occur multiple times, the converted string will have several consecutive repeated characters, which can reduce space storage. The algorithm time complexity of BWT is *O*(*n*^2^).

FM-index is a method based on BWT, which can find the number and position of characters in a string. The complexity of the algorithm is *O*(*n*). In the software of DNA sequence comparison, the advantage of FM-index algorithm is that it can save memory and realize sequence alignment on personal computer.

Suffix tree uses space for time and uses the common prefix of string to reduce the overhead of query time in order to improve efficiency, but it consumes a lot of memory. The algorithm complexity of suffix tree is *O*(*n*), and it also has good performance.

### 1.5. Introduction of Variation Detection Process

Second-generation sequencing technology improves sequencing efficiency and reduces cost, and whole gene sequencing has been realized. Because of the large amount of data generated by sequencing and the complex analysis process, it is necessary to combine a variety of software to analyze the sequencing data. The following documents generated by the sequencing detection process are explained.

#### 1.5.1. Raw Sequencing Data Cleaning

Early gene sequencing tools can only read 100 bases, and, later, according to NGS data of different sequencing platforms, the reading can reach 150–250 bp. Illumina HiSeq 2500 is the world's highest throughput sequencing platform. At present, in about 27 hours, more than 300 billion bases can be measured, and the whole genome and whole exon of 6–7 individuals can be sequenced quickly. Illumina platform uses FastQ format to store sequencing results, and FastQ documents include base read fragments and sequence quality.

In the sequencing process, due to random errors, the original data after sequencing needs to be cleaned before entering the detection process. Taking the sequencing data of tumor gene alignment sequence (SRR12060749) as an example, the preprocessing process is illustrated, and the original sequencing data is filtered. First, clean the single-ended sequencing data, keep the quantity consistent before and after cleaning, and then clean the low-quality data to ensure the reliability of sequencing data before and after cleaning.

It can be seen from Table 2 that the original data of tumor gene alignment sequence sequencing is of high sequencing quality, and the overall data volume after cleaning is as high as 98.83%.

In Table 2, “Clean_len” lists the length of sequences after cleansing, and “Reads” represents the number of sequences sequenced. The purpose of data cleaning is to improve the accuracy and quality of data detection.

The relationship between sequence length and count before and after sequencing data cleaning is shown in Figure 5.

The length of most data before and after sequencing is 75 bp, and the quantity reaches 22 million. The effect of sequencing data quality and quantity distribution before and after cleaning is shown in Figure 6.

As can be seen from Figure 6, the number of sequences with a sequencing quality of 35 reaches 13 million, and most of the sequencing data have a quality above 30. The change of sequencing sequence is seen from the distribution of GC content, as shown in Figure 7.

It can be seen from Figure 7 that the sequencing sequences are basically consistent before and after cleaning, and the GC contents of the two sequences are similar. The relationship between the same test fragments in the sequenced sequence can be seen from the distribution ratio of the repetition degree of the sequenced fragments, as shown in Figure 8.

As can be seen from Figure 9, the proportion of sequencing fragments with repetition of 1 and 2 is relatively large, which is mainly caused by some base variation or machine error in sequencing. The repetitions of sequencing fragments before and after cleaning are similar, and the overall trend is consistent.

The total amount and quality of the sample sequencing data of tumor gene alignment sequence are basically consistent, both at a high level.

#### 1.5.2. Sequencing Sequence Alignment

For more than 60 existing comparison software tools, Bowtie 2, BWA, HISAT2, and Subread are significantly higher in use times and effects than other software tools. The following focuses on the comparative study of these four software tools and the comparative study of the generated BAM files. Take the sequencing samples of tumor gene alignment sequences as an example to illustrate the differences in software alignment effects. The alignment effects are shown in Table 3.

In Table 3, four kinds of sequence alignment software are proposed. Because of the differences in algorithm design and sequence detection, there are differences in detection effect.

According to the statistical results in Table 3, in terms of comparison algorithms, the algorithms adopted by Bowtie 2 and BWA software are based on BWT technology, the algorithms adopted by HISAT2 software are based on FM-index technology, and the algorithms adopted by Subread software are based on hash index technology. In terms of time execution, HISAT2 and Subread take a long time, while Bowtie 2 takes a short time. In terms of sequencing sequence matching efficiency, BWA and HISAT2 have higher matching rates, which are 98.78% and 96.75%, respectively, while Subread and Bowtie 2 have lower matching rates, both of which are lower than 90%. Overall, BWA and HISAT2 software tools have advantages in comparison of rate and time, while Bowtie 2 has poor comparison effect. BWA is a popular comparison software tool at present, which is more suitable for whole gene sequencing and exon sequencing.

As shown in Figure 10, the four types of software are sorted by SAMtools to form BAM files, and it is found that BWA, Bowtie 2, and HISAT2 have the highest number of duplicates (excluding duplicates with other software tools), with the numbers of 492752 and 653738, respectively. The number of duplicates for Bowtie 2 and Subread (excluding duplicates with other software tools) is 21381. BWA, HISAT2 and Subread had a maximum number of duplicates (excluding duplicates with other software tools) of 887,962, while Bowtie 2, HISAT2, and Subread had a maximum number of duplicates (excluding duplicates with other software tools) of 10,371. BWA, HISAT2, Subread, and Bowtie 2 have 11065583 sequence repetitions, which shows that most of the sequencing data are correctly identified.

It is very important to choose the appropriate comparison software to detect SNP, and the speed and accuracy of the comparison software should be considered comprehensively. Therefore, considering the matching rate and comparison quantity of the four comparison software tools, BWA comparison software has certain advantages in detection effect. In the detection of SNP and InDel, BAM files generated by BWA software are used as input files of four variation detection software tools, and the differences between SNP and InDel are further analyzed.

#### 1.5.3. Variation Detection

At present, there are many detection tools for SNP and InDel. Among many detection tools, VarScan 2, GATK, BCFtools, and FreeBayes are widely used. The running platform, input type, output type, and data format of the four software tools are described below, as shown in Table 4.

The Mpileup file is transformed by SAMtools tool after testing the above software. From the software use effect to see the actual situation of various software tools; SNP and InDel are statistically analyzed, as shown in Table 5.

 The above SNP and InDel were filtered (the sequencing depth was greater than 10 and the sequencing quality was greater than 30), which ensured the detection quality. In detecting SNP, FreeBayes has the largest number and VarScan 2 has the least number; in detecting InDel, GATK has the largest number and VarScan 2 has the least number. In terms of overall detection, GATK has the largest number and VarScan 2 has the least number. From the above statistical results, the detection software in the detection of the same sample has a relatively large difference, which is due to the use of detection technology caused by this difference. The differences in the numbers of SNP and InDel detected by the four detection software tools are shown in Figures 9 and 11.

In Figure 12, the same number of SNP detected by the four software tools is 23157, indicating that most SNP variation points are detected by all four software tools. BCFtools, FreeBayes, and GATK have high similarity in detecting SNP and share more variation points. Four kinds of software detected the same number of 795 on InDel, GATK detected the largest number, and the other three kinds of software were similar in number.

#### 1.5.4. Sequencing Data Variation Detection Process

The data processing flow begins with reading sequence alignment (BWA [16]), followed by raw data cleansing (Picard [17]), sequence recalibration, filtering, variable invocation, recalibration (GATK [18]), coverage analysis (BedTools [19]), and annotation (Annovar [20] and internal annotation tools). This process requires a combination of biological software with additional comments and override steps. Generally speaking, the analysis process includes three key stages: (1) preparing the original sequence for variation discovery and coverage calculation, (2) variation call and recalibration; and (3) variation filtering and annotation. The sequence data variation detection process is shown in Figure 12.

In Figure 12, the whole process from planetary sequence sequencing to mutation annotation is mainly used to explain the sequencing workflow in detail. Each link is the key work of the research, which can clearly reflect the research focus of each stage of the research work.

## 2. Method

### 2.1. Variant Expression of Sparse DNA Sequence

Sparse theory is used to detect variation points in DNA sequences, and SNP and InDel variation account for less than 0.1% of DNA sequences. In this way, SNP and InDel variations show the sparsity of the whole sequence compared with the whole DNA sequence or exon sequence. Therefore, the exons are used as the basis of the matrix, and the variation points in the matrix are used as marks 1.

In DNA sequences or exon sequences, the core of sparse representation is the solution of linear equations *y* = Ax, where matrices *A* ∈ *m* × *n* and *A* are usually full rank. *M* denotes the number of DNA or exon sequences, and *N* denotes the variation point variable. In a given *m*-dimensional space, a set of overcomplete bases *A* ∈ *m* × *n* can be sparsely represented by selecting the least number of basis vectors *y* ∈ *m*, and its strict definition can be expressed as

(4) $$\begin{array}{c} \min{\left\|x\right\|}_{0}\text{s}.\text{t}.y=Ax. \end{array}$$

If matrix *A* satisfies the condition

(5) $$\begin{array}{c} \sigma \left(A\right)\geq 2{\left\|x\right\|}_{0}, \end{array}$$

where *σ*(*A*) refers to the number of vectors contained in the minimum linearly correlated column vector set, then the *L*0-norm optimization problem in formula (4) has a unique solution.

It is difficult to solve the linear equation *y*, and the *L*0-norm optimization problem has the same solution as the *L*1-problem; namely,

(6) $$\begin{array}{c} \min{\left\|x\right\|}_{1}\text{ s}.\text{t}.\;y=Ax. \end{array}$$

The finite equidistant property condition is a measure of the orthogonality of a column vector; that is, it has a constant *μN* that satisfies certain conditions:

(7) $$\begin{array}{c} \left(1-\mu N\right){\left\|x\right\|}_{2}^{2}\leq {\left\|Ax\right\|}_{2}^{2}\leq \mu N{\left\|x\right\|}_{2}^{2},\;\forall x,{\left\|x\right\|}_{0}\leq N. \end{array}$$

Due to the presence of noise *ε*, the sparse expression is optimized. If formula (8) is satisfied, the optimization condition is satisfied.

(8) $$\begin{array}{c} \min{\left\|x\right\|}_{0}\text{ s}.\text{t}.{\left\|y-Ax\right\|}_{2}^{2}\leq \varepsilon . \end{array}$$

If there are samples of different classes of tags in the DNA sequence expression matrix, the sample tags in the divergence matrix are passed. The divergence matrix is divided into the following:

(9) $$\begin{array}{c} \left\{\begin{array}{c} S_{b}=\overset{c}{\underset{j=1}{\sum }}N_{j}\left(\mu_{j}-\mu \right){\left(\mu_{j}-\mu \right)}^{T},\\ S_{w}=\overset{c}{\underset{j=1}{\sum }}\overset{N_{j}}{\underset{i=1}{\sum }}\left(x_{i}^{j}-\mu_{j}\right){\left(x_{i}^{j}-\mu_{j}\right)}^{T},\\ S_{t}=S_{b}-\eta S_{w}. \end{array}\right. \end{array}$$

Here, *S*_*b*_ and *S*_*w*_ represent interclass divergence matrix and intraclass divergence matrix, respectively, and represent adjustment parameters.

The distances between classes and within classes can be calculated by using the trace of the corresponding divergence matrix, and their calculation formula is

(10) $$\begin{array}{c} \left\{\begin{array}{c} \text{trace}\left(S_{b}\right)=\text{trace}\left[\overset{c}{\underset{j=1}{\sum }}N_{j}\left(\mu_{j}-\mu \right){\left(\mu_{j}-\mu \right)}^{T}\right]=\lambda_{b1}+\lambda_{b2}+\cdots +\lambda_{bk},\\ \text{trace}\left(S_{w}\right)=\text{trace}\left[\overset{c}{\underset{j=1}{\sum }}\overset{N_{j}}{\underset{i=1}{\sum }}\left(x_{i}^{j}-\mu_{j}\right){\left(x_{i}^{j}-\mu_{j}\right)}^{T}\right]=\lambda_{w1}+\lambda_{w2}+\cdots +\lambda_{wk}. \end{array}\right. \end{array}$$

*η* can be expressed by the ratio in formula (10):

(11) $$\begin{array}{c} \eta =\frac{\text{trace}\left(S_{b}\right)}{\text{tarce}\left(S_{w}\right)}. \end{array}$$

In formulas (10) and (11), *S*_*b*_ represents the divergence matrix between classes and the divergence matrix in different regions of SNP and InDel; *S*_*w*_ represents the total divergence matrix, representing the divergence matrix in all regions of SNP and InDel; “trace” represents the separation of distance between measured sample classes, which is used to describe the separation of SNP and InDel variants. *η* is used to evaluate the proportion relationship in different regions and describe the ratio of SNP and InDel variation in different regions.

### 2.2. Bayesian Statistics

#### 2.2.1. Conditional Probability

Considering the correlation with event *A*, when the probability of occurrence of event *B* is recorded, it is called the conditional probability (posterior probability) of occurrence of event *B* on the basis of occurrence of event *P*(*B|A*). Similarly, *P*(*A*) is called unconditional probability (prior probability). It can be described by the following formula:

(12) $$\begin{array}{c} P\left(B|A\right)=\frac{P\left(\text{AB}\right)}{P\left(B\right)}. \end{array}$$

If *A* and *B* are two arbitrary nonzero events, the probability of their product is equal to the product of the conditional probability of the occurrence of event *B* or event *A* when *A* occurs or *B* also occurs.

(13) $$\begin{array}{c} \left\{\begin{array}{c} P\left(A\cdot B\right)=P\left(A\right)\cdot P\left(B|A\right),\\ P\left(A\cdot B\right)=P\left(B\right)\cdot P\left(A|B\right). \end{array}\right. \end{array}$$

If *A* and *B* are incompatible events, the product is equal to the product of the probabilities of *A* and *B* as follows:

(14) $$\begin{array}{c} \left\{\begin{array}{c} P\left(A\cdot B\right)=P\left(A\right)\cdot P\left(B\right),\\ P\left(A\cdot B\right)=P\left(B\right)\cdot P\left(A\right). \end{array}\right. \end{array}$$

If three or more events occur, product *P*(*A*_1_*A*_2_,…, *A*_*n*−1_) > 0 of *n* events can be described by the following equation:

(15) $$\begin{array}{c} P\left(A_{1}A_{2}\ldots A_{n}\right)=P\left(A_{n}|A_{1}A_{2}\ldots A_{n-1}\right)P\left(A_{n-1}|A_{1}A_{2}\cdots A_{n-2}\right)\ldots P\left(A_{2}|A_{1}\right)P\left(A_{1}\right). \end{array}$$

If *n* events are independent of each other, they are described as

(16) $$\begin{array}{c} P\left(A_{1}A_{2}\cdots A_{n}\right)=P\left(A_{n}\right)P\left(A_{n-1}\right)\cdots P\left(A_{2}\right)P\left(A_{1}\right). \end{array}$$

If, for all sample spaces, *B* is an event in sample space, *A*_1_*A*_2_ … *A*_*n*_ are all factors affecting *B*; it is called a complete event in sample space, and *P*(*B*_*i*_) > 0 (*i*=1,2,…, *n*) is described as *P*(*B*):

(17) $$\begin{array}{c} P\left(B\right)=P\left(B|A_{1}\right)P\left(A_{1}\right)+P\left(B|A_{2}\right)P\left(A_{2}\right)+\cdots +P\left(B|A_{n}\right)P\left(A_{n}\right)=\overset{n}{\underset{j=1}{\sum }}P\left(A|B_{i}\right)P\left(B_{i}\right). \end{array}$$

If, for all sample spaces, *B* is an event in sample space, *A*_1_*A*_2_ ⋯ *A*_*n*_ are all factors affecting *B*, which is called a complete event in sample space, and *P*(*B*) > 0, *P*(*A*_*i*_) > 0(*i*=1,2,…, *n*) can be described as

(18) $$\begin{array}{c} P\left(A_{i}|B\right)=\frac{P\left(B|A_{i}\right)P\left(A_{i}\right)}{\sum_{j=1}^{n}P\left(B|A_{j}\right)P\left(A_{j}\right)}, \end{array}$$

(19) $$\begin{array}{c} \overset{n}{\underset{j=1}{\sum }}P\left(B|A_{j}\right)P\left(A_{j}\right)=\overset{n}{\underset{j=1}{\sum }}P\left(B,A_{j}\right)=P\left(B\right). \end{array}$$

And ∑_*j*=1_^*n*^*P*(*A*_*j*_)=1 and *P*(*A*_*j*_) represent the probability of event *A*_1_*A*_2_ … *A*_*n*_, which is the prior probability of assuming event *P*(*A*_*i*_*|B*). EE says that if event *B* occurs, it assumes a posterior probability of event *A*_1_.

#### 2.2.2. Bayesian Reasoning in Data Fusion

Bayesian reasoning realizes the fusion of BAM files compared by multiple DNA sequence alignment software tools. To calculate the posterior probability when a given condition occurs [21, 22], set *n* comparison software tools to sequence the same original sequencing file. Assume that there are *m* alignment sequences in the original sequencing which need to be aligned and identified; that is, there are *m* hypotheses or propositions *A*_*i*_,  *i*=1,2,…, *m*. Specifically through multilevel classification in the first level, identify the information features obtained from the original sequencing data and classify the attributes, obtain the target attributes *B*_1_, *B*_2_,…, *B*_*n*_, calculate the likelihood function of each comparison software tool under each hypothesis according to the correct classification of sequencing data and comparison, calculate the posterior probability of each hypothesis under multiple comparison lines of evidence according to Bayesian inference, and finally generate the attribute judgment conclusion according to the judgment logic. The process is shown in Figure 13.

There are two steps in calculating the fusion probability of alignment sequence. The first step is to calculate the combined likelihood probability function of *n* lines of evidence under the assumption that *A*_*i*_ holds. When each comparison software tool sequences independently and *B*_1_, *B*_2_,…, *B*_*n*_ are independent of each other, the combined likelihood probability distribution is as follows:

(20) $$\begin{array}{c} P\left(B_{1},B_{2},\ldots ,B_{n}|A_{j}\right)=P\left(B_{1}|A_{j}\right)P\left(\left.B_{2}\right\}A_{j}\right)\cdots P\left(B_{n}|A_{j}\right). \end{array}$$

Then, using Bayesian formula, the posterior probability of *A*_*j*_ under the condition of *n* lines of evidence is obtained.

(21) $$\begin{array}{c} P\left(A_{j}|B_{1},B_{2},\ldots ,B_{n}\right)=\frac{P\left(B_{1},B_{2},\ldots ,B_{n}|A_{j}\right)P\left(A_{j}\right)}{P\left(B_{1},B_{2},\ldots ,B_{n}\right)}. \end{array}$$

In the reasoning process of Bayesian combinatorial logic, the maximum a posteriori probability reasoning logic is used to directly use the target attribute of the decision threshold maximum a posteriori combination joint probability. Select the formula that meets *A*_*i*_ condition:

(22) $$\begin{array}{c} P\left(A_{j}|B_{1},B_{2},\ldots ,B_{n}\right)=\underset{1\leq j<n}{\max}P\left(A_{j}|B_{1},B_{2},\ldots ,B_{n}\right). \end{array}$$

According to the above formula, the decision threshold is established in the assumption of maximum a posteriori probability, and the decision threshold of specific rule *A*_*j*_ is established.

(23) $$\begin{array}{c} P\left(A_{j}|B_{1},B_{2},\ldots ,B_{n}\right)\geq P_{o}. \end{array}$$

If *A*_*j*_ is accepted, reject it, determine the next rule, form new evidence, and then determine the above way [23].

### 2.3. Research on Multi-Information-Based Data Fusion

#### 2.3.1. Data Fusion of Sequencing Sequence Alignment

The purpose of this study is to improve the success rate of comparison, and different comparison software tools may lead to comparison effect. In order to improve the effect of comparison and find more structural variations, this paper adopts data fusion based on multicomparison software. Its multicomparison software comparison data fusion process is shown in Figure 14.

In the above process, the Sort part adopts the condition of counting the sequences in SAM file, counts the number of sequences, and sorts them according to the number. The four tools are sorted after the sequence comparison, for the same sequence appears in all the files, indicating that the sequence alignment is correct. If the same sequence appears in three files and the frequency of sequence occurrence is quite high, it also indicates that the sequence alignment is correct. If the same sequence appears in two files and the frequency of sequence occurrence is quite high, refer to PCR sequence. If the PCR sequence is in the target sequence, the alignment is correct; in other cases, the sequence can be deleted or ignored as an alignment result. Gene sequences are compared by the above four software tools, and then the post-SAM files are sorted to form BAM files. The following is the comparison algorithm shown in BAM file in Algorithm 1.

#### 2.3.2. Research on SNP Calling Data Reasoning

In the process of sequencing, SNP has a great correlation with many diseases, and more SNP are found in order to find out the correlation analysis between variation points and diseases [24, 25]. There are some differences in finding SNP among the above four kinds of software, which are mainly caused by the differences in algorithm design adopted by the software itself. Therefore, this paper proposes merging the above four tools in order to count more SNP, and its structural flow is shown in Figure 15.

After the above four tools form VCF files, they are merged to remove duplicate data. Then, through the filtering mechanism in GATK [26], the recommendation mechanism in SNP and InDel is analyzed, and finally the filtered VCF is generated and then annotated by annotation software. The inference mechanism and sequence alignment in the SNP Calling process are too similar to each other and will not be described here.

## 3. Results

### 3.1. Comparison of Experimental Results

This paper compares the above four software tools Bowtie 2, BWA, HISAT2, and Subread. In the comparison part of SNP and InDel, we use GATK, BCFtools, FreeBayes, and VarScan 2 to detect SNP and InDel variation. The main research work of this part is to analyze the points of variation detection and then perform comparison with the fusion method of recommendation mechanism.

In the experiment, SVsim software is used to simulate the DNA data of double-end sequencing, and the corresponding error rate, sequencing length, and sequencing type are set. 3000 SNP sites and 2000 InDel sites (2–10 bp insertion, 2–10 bp deletion) were inserted into the simulated sequencing sequence. Six Illumina simulation samples were generated by sequence simulation software, and the test depths were 50, 100, 150, 200, 250, and 300, respectively. The standard error and error rate of sequencing were 0.

This paper takes cancer gene test data as the research object and compares the sequence number of software and reasoning fusion methods from different test depths, as shown in Figure 16.

When comparing the number of SNP and InDel, the correctness of software detection cannot be guaranteed by comparing the actual data, and different software tools will produce different comparison when testing the same data. Therefore, in this paper, 3000 SNP and 2000 InDel variation points are inserted into the test data, and this fixed variation point is taken as the comparison object. With the increase of different test depths, the variation detection points also increase, as shown in Figures 17 and 18.

As can be seen from Figures 19 and 20, with the increasing test depth, the number of SNP and InDel variation detections of the test sequence also increases. It shows that increasing the test depth can increase the number of variation detections in the test work.

### 3.2. Performance Analysis

In the process of DNA cancer gene test data, the sequencing results of GATK, Bcftools, Freebayes, and VarScans in the BAM file are fused by the Bayesian model. The mutation site sensitivity estimate is described [26] in terms of recall as follows:

(24) $$\begin{array}{c} \text{Recall}=\frac{\text{TP}}{\text{TP}+\text{FN}}. \end{array}$$

As can be seen from Figures 19 and 20, due to the increased sequencing depth found in SNP and InDel, it is shown that there is enough sequencing depth in the sequencing data to ensure the correctness and recall rate of SNP and InDel. In the sequencing process, there can be enough sequencing depth and high accuracy.

As can be seen from Tables 6 and 7, at runtime, GATK, BCFtools, FreeBayes, and VarScan 2 need to be made into BAM files by BWA software, which takes a certain amount of time. However, the reasoning method proposed in this paper is based on the above methods, which takes up more time. Besides BWA, the running time of GATK is also long, which is limited by software algorithm. But the effect of GATK is also ideal. With the increase of sequence length, the accuracy and recall rate of the proposed method also increase, and, with the increase of sequence length, the comparison time also increases, so the running time also increases.

## 4. Conclusion

In the era of rapid development of second-generation sequencing, it has become an important direction of medical development to establish the relationship between gene variation and diseases by DNA sequencing. In this paper, SNP and InDel detection methods based on machine learning and sparse matrix detection are proposed, and VarScan 2, GATK, BCFtools, and FreeBayes are compared. In the research of SNP and InDel detection with intelligent reasoning, the experimental results show that the detection accuracy and recall rate are better when the depth is increasing. The reasoning fusion method proposed in this paper has certain advantages in comparison effect and discovery in SNP and InDel and has good effect in swelling and pain gene detection. In this paper, different software detection methods are studied for fusion. After fusion, there are obvious advantages in the number of SNP and InDel. However, in the case of large-area sequence missing, the detection effect is poor, so it is necessary to further reason and fuse the detected sequence position information. The later work mainly focuses on the selection of sequences after fusion and studies the characteristics of sequences, so that different software fusion can be selected to achieve the best performance.

## Figures and Tables

**Figure 1:** BWT transformation process.

**Figure 2:** Suffix tree of *S*.

**Figure 3:** Suffix array of *S*.

**Figure 4:** FM-index transformation process.

**Figure 5:** The relationship between sequence length and count before and after cleaning.

**Figure 6:** The relationship between sequence quality and count before and after cleaning.

**Figure 7:** Sequence GC distribution before and after cleaning.

**Figure 8:** Distribution ratio of sequenced duplication level.

**Figure 9:** Comparison of differences between detection software tools in SNP.

**Figure 10:** Comparison of repeated quantity of four alignment software tools.

**Figure 11:** Comparison of differences between detection software tools in InDel.

**Figure 12:** Flow chart of variation detection of sequencing data.

**Figure 13:** Sequence fusion based on Bayesian inference.

**Figure 14:** Data fusion process under intelligent reasoning.

**Figure 15:** SNP and InDel convergence process.

**Figure 16:** Comparison between this method and other methods.

**Figure 17:** SNP detection quantity comparison.

**Figure 18:** Comparison of SNP detection quantity.

**Figure 19:** SNP recall rate of detection software.

**Figure 20:** InDel recall rate of detection software.

**Algorithm 1:** Fusion reasoning algorithm flow.

**Table 1:** Hash table of sequence *S* (*k* = 2).

Seed	*V*(*w*)	Position	Seed	*V*(*w*)	Position	Seed	*V*(*w*)	Position

AA	0	(1, 7) (1, 8)	CG	6	(1, 2)	GT	11	(1, 3)
AC	1	(1, 1) (1, 5)	CT	7		TA	12	(1, 4)
AG	2		GA	8		TC	13	
AT	3	(1, 9)	GC	9		TG	14	
CA	4	(1, 6)	GG	10		TT	15	
CC	5							

**Table 2:** Comparison before and after data cleaning.

Sample	Len	Clean_len	Reads	Clean_reads	GC %	Rate %

SRR12060749_1	1–75	20–75	23389073	23115063	49	98.828
SRR12060749_2	1–75	20–75	23388231	23115063	49	98.832

**Table 3:** Comparison of four software sequences.

Soft	Algorithm	Mapped	Total	Mapped rate (%)	Time (s)

Bowtie 2	BWT	40499908	46230126	87.61	1316
BWA	BWT	47650174	48239938	98.78	1549
HISAT2	FM-index	52138360	53891457	96.75	2111
Subread	Hash index	41308336	46230126	89.35	2694

**Table 4:** Comparison of parameters of four variation detection tools.

Soft	System	Input	Output	Identifies

GATK	Lin	SAM/BAM	VCF	SNP, InDel
BCFtools	Lin	SAM/BAM	VCF	SNP, InDel
FreeBayes	Lin	SAM/BAM	VCF	SNP, InDel
VarScan 2	Lin, Mac, Win	Mpileup	VCF, CSV	SNP, InDel, CNV

**Table 5:** Number of SNP and InDel.

Soft	SNP	InDel	Total

GATK	48084	15391	63475
BCFtools	53255	3710	56965
FreeBayes	53549	4671	58220
VarScan 2	29588	2200	31788

**Table 6:** SNP accuracy of detection software.

Soft	50×	100×	150×	200×	250×	300×

GATK	75.13%	77.47%	81.70%	84.53%	88.47%	94.83%
BCFtools	70.47%	74.40%	76.30%	78.83%	81.80%	85.50%
FreeBayes	67.70%	71.80%	74.03%	76.70%	78.47%	81.90%
VarScan 2	71.90%	75.50%	77.47%	79.57%	84.90%	88.47%
Our method	73.83%	77.37%	80.13%	84.53%	93.37%	97.43%

**Table 7:** Checking the correct rate of software InDel.

Soft	50×	100×	150×	200×	250×	300×

GATK	67.80%	71.20%	74.35%	77.90%	81.20%	87.90%
BCFtools	64.45%	67.70%	69.85%	72.30%	77.35%	81.80%
FreeBayes	60.70%	64.90%	66.75%	69.35%	74.90%	80.05%
VarScan 2	63.90%	68.40%	70.20%	73.70%	78.40%	84.85%
Our method	70.50%	76.35%	79.90%	83.35%	89.85%	96.15%

## Data Availability

The experimental data used to support the findings of this study are available from the corresponding author upon request.
